# The Immune Infiltration in HNSCC and Its Clinical Value: A Comprehensive Study Based on the TCGA and GEO Databases

**DOI:** 10.1155/2021/1163250

**Published:** 2021-11-08

**Authors:** Xizhe Sun, Lijia Zhang, Songjiang Liu

**Affiliations:** ^1^Heilongjiang University of Chinese Medicine, China; ^2^First Affiliated Hospital, Heilongjiang University of Chinese Medicine, China

## Abstract

**Background:**

Being potential field of research for tumor immunological therapy, the head and neck squamous cell carcinoma (HNSCC) is one of most discussed types of tumor. Recently, some clinical trials have also used immunological therapy and demonstrated a subset of HNSCC patients who have shown a clear longer survival time.

**Objective:**

To conduct further studies and deeper research in the immunological oncology of HNSCC, a more detailed description and comprehending of the complicated landscape of immune infiltrative may be required.

**Methods:**

Firstly, we have described the fraction of different infiltrating immune cells in the HNSCC tumor and then compared it to the normal tissue, and secondly, we have explored the clinical implications of various infiltrated immune cell fractions meticulously. The gene expression profiles of HNSCC tissue were obtained from databases of TCGA and GEO and utilized the deconvolution algorithm (CIBERSORT) to presume the fractions of 22 several immune sensitive cells.

**Results:**

Our results indicated that the immune infiltrating cell fractions were considerably different between HNSCC tumor tissue and paired normal tissue, but at the same time, we found a potential internal correlation among the immune cells and also showed the association between immune infiltrating cells and their clinical characteristics. It is worth noting that the resting dendritic cells and M1 macrophages were linked with a favorable prognosis, while the CD4+ T cells with a poorer outcome.

**Conclusion:**

Fractions of immune cell percentage were also associated with tumors' pathological grade, age, and TNM stage.

## 1. Introduction

Every year, 600,000 subjects are being diagnosed with HNSCC in the world. It is reported as the common cancer ranked as sixth with 40% to 50% of a mortality rate [1–4]. As we know, the most common therapy method used previously and currently for HNSCC is aimed at reducing its toxicity and lowering the morbidity rate. However, recurrent diseases and metastatic tumors are usually considered incurable and also show a poor prognosis. Therefore, more effective therapies are needed to be explored in patients with advanced HNSCC, for example, target therapies. However, despite a 10% to 15% response rate of the single-drug therapy cetuximab, we admit being unaware of any biomarkers that are found effective to date [5, 6].

In traditional research on malignant carcinoma target therapy, the molecular pathways seem to be too complex for comprehensive understanding by some researchers. Although another potential therapy, namely, immune therapy may potentially avoid this drawback, it is argued by some current studies [7, 8]. Despite most of the HNSCC patients being resistant to immune therapy, some patients could be benefitted from it and may display a better prognosis with less toxicity. Though the precise reason and the mechanistic basis remains unclear, the consequence that occurs could be a result of the related factors present, e.g., deficient immune surveillance, a deficient of proper rejection antigens, or immune-suppressive mediators presence in the HNSCC tumor microenvironment [9]. Also, the fraction of immune cell infiltration was proved to have an important role in human malignant tumors and was associated with patients' survival, thus, acting as a potential biomarker [10]. To further explore the immuno-oncology diagnosis and treatment for HNSCC, a particular understanding of the landscape of infiltrating fraction of the immune cells may be required, along with an understanding of the effect of these factors on the clinical consequence [9].

We explored the data from the GEO and TCGA databases and then comprehensively summarized and compared the immune cell infiltrating fraction landscape between HNSCC patients' tissues and normal tissues. Also, we investigated its relationship with patients' survival. Our description of the HNSCC-infiltrative immune cell landscape may help in guiding the clinical investigation within immunooncology.

## 2. Materials and Methods

### 2.1. Sample Collection

The samples for study were obtained from databases of “The Cancer Genome Atlas (TCGA)” and “the Gene Expression Omnibus (GEO)”. The relevant data and expression profiles of gene in the clinical data of HNSCC were updated on the 31st of December 2018 in the two public datasets, which were further downloaded and explored [11, 12]. In the GEO database, the duplicate and small sample size (*n* < 50) datasets were excluded, and the verification was performed by two people to maintain accuracy. In the TCGA datasets, the preprocess and the resultant raw data were used in a multiarray average algorithm. For transformation of RNA sequencing data, variance modeling was utilized at the observational level (voom), which induces similarities in microarray-obtained sequencing data. [13]. Next, we changed all the gene probe names to the relevant gene names according to the platform annotation files. Then, we put in every unit and related clinical data for further analysis and distinguished between tumor tissue and normal tissue manually. Later, we screened the significantly different immune infiltrating cells and aimed to study the difference between the infiltrated cells in HNSCC cancer as well as normal tissue.

### 2.2. The Number of Tumor-Infiltrating Immune Cells

For gene expression profiles and its analysis, CIBERSORT is a highly applicable analytical tool that analyzed 547 genes. A deconvolution algorithm was used to describe each subtype of immune cell and quantify precisely certain immune cell. A decreased *P* value exhibited low degree of relationships among types of immune cells statistically and traced out samples with low accuracy.

Once the primary gene expression data was obtained, a change had to be performed to further run CIBERSORT as previously reported by Chen et al. [14]. The CIBERSORT (http://cibersort.stanford.edu) was a database on which obtained information was analyzed at the permutation number of 100. The correlation ratios were also evaluated among 22 types of infiltrating immune cells, and each analyzed with CIBERSORT indicators such as the value of *P* (Pearson's correlation coefficient) and the root mean square error (RMSE).

### 2.3. Statistical Analysis

For the samples to be analyzed, the CIBERSORT *P* value had to be <0.05. The Pearson's correlation coefficient was used to evaluate relationships between all types of immune cells. The Kruskal-Wallis or Wilcoxon test was applied to analyze the relationship among categorical and continuous variables. Keeping the median value of the immune cell ratios, the survival analysis was performed for each cell subtype. For contrasting survival curves among different types of patient's groups, the Log-rank Mantel-Cox regression was performed, while regression was performed using GraphPad Prism 7.0 software. Furthermore, based on gender, age, histological grade, status of lymphocytes, and TNM stage, SPSS 24.0 was used to adjust the multivariable analysis.

Overall statistical analysis was two tailed. The test with significance is with *P* value < 0.05. The R version 3.6.2 was used to complete all analyses.

## 3. Results

### 3.1. The Landscape of Immune Infiltration in HNSCC

Table 1 shows the landscape of infiltration of 22 immune cell fractions and distinguishes tumor tissue from paired normal tissue in HNSCC. A contrasting result can be seen in the percentage of immune cells among both groups (Figure 1). The HNSCC tumor tissue contained a larger number of CD8+ T cells, M0 macrophages, resting NK cells, and dendritic cells compared to the paired normal tissue. However, plasma cells, regulatory T cells (Tregs), monocytes, and neutrophils were found to be relatively lower (Figure 2(a)). The ratios of 22 tumor-infiltrative immune cells (TIICs) were found to be more or less correlated to the tumor. The naïve CD4 memory T cells and B cells exhibited the most positive correlation (Pearson′s correlation = 0.62). Moreover, resting CD4+ memory plasma cells and T cells exhibited negative correlation, but the monocytes and CD8+ T cells were also found to be positively correlated due to Pearson's correlation value of 0.62 (Pearson′s correlation = 0.69) (Figures 2(b) and 2(c)). Overall, the conclusions suggested that the immune response of HNSCC indicated a complicated network with a continued rigid way of adjusting and controlling.

### 3.2. The Clinical Implications of TIIC Subsets

The GEO datasets did not reveal about survival rates. So, the data of HNSCC as exhibited by statistical relationship among the overall survival and the specific TIICs were obtained TCGA and analyzed through the univariate Cox regression via GraphPad Prism 7.0. However, we obtained 102 subjects with overall survival data after limiting the CIBERSORT filter to *P* < 0.05. The unadjusted HRs, detailed 95% CI, and the *P* value for the median fractions of subtypes of TIICs are displayed in Table 2, while the relevant Kaplan-Meier curve and Log-rank test are displayed in Figure 3.

Further, we identified the relationship among various immune cell types and then explored the relationship of these immune cell types with the pathological grade, age, and TNM stage of HNSCC by settling the features with the pathological information from databases of TCGA and GEO. We extracted the final report of pathological grading that exhibited varied percentages of helper follicular T cells, CD8 T cells, M1 macrophages, and neutrophils. The percentage of follicular helper T cells is varying factor with age which may increase in older individuals. The ratio of M0 macrophages was linked to the T stage, while the regulatory T cell (Tregs) fraction was associated with the N stage (Figure 4).

## 4. Discussion

The tumor microenvironment includes cells of malignant carcinoma, different kinds of immune infiltrating cells, fibroblasts, cytokines, and chemokines and is a complicated biological process. It is also regarded as a dynamic ecosystem with a complex internal structure. This intricate ecosystem has acquired wide attention from oncologists. The researchers have reported that the function of the immune response in this ecosystem is to regulate the action of tumor growth and invasion and eventually lead to metastasis of the tumor. Therefore, it is regarded as another possible target for therapy except in cases, where traditional treatment strategies are used, such as chemotherapy and radiation therapy [15]. According to some published studies, immune therapy has shown good clinical results in several other types of malignant tumors. However, still, many patients do not benefit or show only a little response to the same regimen. In the case of HNSCC, the current situation of immune therapy does not show any improvement compared to other tumor types, and we are also not aware of the patients who could benefit from it [16]. However, compared to other malignant tumors, HNSCC patients are expected to benefit from immune therapy currently. The approach and results to date are largely experience-based and do not have much evidence available. Our data reminds us to pay attention to the immune checkpoint blockade and also discover the pattern of success from previous successful clinical cases. For further detailed clinical research on HNSCC, deeper comprehension of the immune landscape is required.

Here, we used public databases and analyzed the immune infiltration in HNSCC and further explored the influence of these attributes on clinical consequences. The development of computing means has led to the discovery of CIBERSORT, which is a deconvolution algorithm that can analyze data from carcinoma transcriptomes. We utilized it for extraction of fractions of 22 tumor-infiltrating cells. This method was successfully used in breast cancer and lung cancer and was confirmed by FACS [17, 18]. Thus, we used CIBERSORT to figure out different patterns of immune infiltrating cells in HNSCC and also discovered the relationship of different immune cell fractions with the clinical prognosis and traits.

The results indicated obvious contrasts in the immune cell proportion between HNSCC and the normal tissue. Our study showed that compared to the normal tissue, HNSCC tissue bears a large number of the following cells: CD8+ T cells, resting NK cells, M0 macrophages, and activated dendritic cells. However, plasma cells, regulatory T cells (Tregs), monocytes, and neutrophils were relatively lower. Furthermore, naïve memory CD4 T cells and B cells, along with monocytes and CD8+ T cells, showed the strongest positive correlation, while plasma cells and CD4+ resting memory T cells exhibited the most obvious negative association. It is reported that CD8+ T cells can identify certain antigens on tumor cells and have significant role in controlling cancer [19]. High fractions of infiltrated CD8+ T cells were exhibited to be linked with diagnosis/screening in quite a majority of cancers [20], aiming to recover the immune response mediated by T cells, for which, many immune therapy regimens in different forms were designed and attempted [16]. NK cells also contribute in the immune response by regulating inhibitory receptors. Several kinds of receptors were also related to the autoimmune activity mediated by NK cells, such as T cell Ig mucin receptor 3, and the lymphocyte activation gene. The inhibiting function of these factors on the NK cells has been reported by some scholars [21, 22]. HNSCC is a sort of malignant tumor that features a significantly high quantity of NK cell infiltration in the immune microenvironment. Thus, researchers have hypothesized that some HNSCC patients may benefit from blocking these receptors [9].

Our clinical analysis exhibited that a higher portion of resting NK cells and M1 macrophages, along with a lower portion of CD4+ lymphocyte were linked to good overall survival. Further analysis on clinical characteristics revealed that the modifications in the ratio of M1 macrophages, neutrophils, CD8+, and follicular helper lymphocyte were associated with the pathological grade of the tumor and increase with patient's age. The percentage of M0 macrophages was interrelated with the T stage, while the regulatory T cell (Tregs) fraction was linked to the N stage. Although several trials have evaluated the predicting significance of CD4+ lymphocyte infiltration in HNSCC, its exact assignment in the tumor microenvironment remains unclear [23]. In the tumor immune infiltrating microenvironment, a large amount of CD4+ cell subtypes are present, which perform various functions, e.g., they stimulate Th1 cells and inhibit regulatory T cells. Thus, scholars have paid attention to stain CD4 expression only but have also attached importance to different subsets [24, 25]. A recent meta-analysis [26], including four studies on CD4+ T cells, suggested that a higher CD4+ TIL infiltration could act as a biomarker, presenting a better survival rate for HNSCC patients. However, the study also argued that it was impossible to obtain the data from most of the research that was concerned with the predicting value of CD4+ lymphocytes. Also, the researchers admitted that due to the lack of statistical significance, some studies did not report negative results, leading to a probable publication bias. Hence, the number of studies discussing the function of CD4+ lymphocytes was found to be relatively lower and not very persuasive. We are, therefore, not sure of the potential prognostic value of CD4+ lymphocytes, and more studies are needed to be designed and implemented in the future.

## 5. Conclusion

Immunotherapies are developing at an unprecedented speed and are also applied in various carcinoma types. Soon enough, immunotherapy may be performed in the standard and normative therapy regimens in HNSCC patients [27, 28].

## Figures and Tables

**Figure 1:** The perspective of immune infiltration with differences in HNSCC. (a) GEO database; (b) TCGA database.

**Figure 2:** (a) Violin plot envisaging the differentially infiltrated immune cells; (b) heatmap of correlation among infiltrated immune cells in tumor; (c) heatmap of the 22 immune cell.

**Figure 3:** Survival plots of median of immune cell fractions.

**Figure 4:** Correlation of distinct immune cell proportions with clinical attributes in HNSCC.

**Table 1:** Comparison of 22 TIIC proportions between the HNSCC tissue and paired normal tissue.

Cell type	CIBERSORT fraction in % (mean ± SD)		
	Paired normal tissue	Tumor tissue	*P* value
B cells			
Naïve	0.021 ± 0.022	0.014 ± 0.027	0.219
Memory	0.034 ± 0.067	0.014 ± 0.041	0.06
T cells			
CD8	0.104 ± 0.057	0.095 ± 0.089	0.646
CD4 naïve	0.163 ± 0.052	0.084 ± 0.072	**<0.001**
Memory resting CD4	0.011 ± 0.037	0.002 ± 0.01	**0.015**
Memory-activated CD4	0.128 ± 0.088	0.131 ± 0.08	0.878
Follicular helper	0.012 ± 0.022	0.033 ± 0.033	**0.005**
Regulatory (Tregs)	0.007 ± 0.013	0.03 ± 0.032	**0.001**
Gamma delta	0.041 ± 0.045	0.028 ± 0.028	0.065
NK cells			
Resting	0 ± 0	0.003 ± 0.01	0.162
Activated	0.023 ± 0.025	0.028 ± 0.028	0.444
Monocytes	0.037 ± 0.032	0.015 ± 0.022	**<0.001**
**Macrophages**			
M0	0.12 ± 0.063	0.015 ± 0.03	**<0.001**
M1	0.012 ± 0.022	0.202 ± 0.138	**<0.001**
M2	0.009 ± 0.028	0.072 ± 0.06	**<0.001**
Dendritic cells			
Resting	0.107 ± 0.105	0.09 ± 0.052	0.224
Activated	0.015 ± 0.03	0.034 ± 0.05	0.071
Mast cells			
Resting	0.041 ± 0.033	0.039 ± 0.042	0.821
Activated	0.071 ± 0.043	0.032 ± 0.04	**<0.001**
Plasma cells	0.006 ± 0.016	0.022 ± 0.04	**0.049**
Eosinophils	—	0.001 ± 0.011	0.513
Neutrophils	0.037 ± 0.067	0.015 ± 0.027	**0.006**

The significance is shown in bold fonts at *P* < 0.05.

**Table 2:** A prognostic association among the subpopulations of 22 TIICs.

Tumor-infiltrating immune cells	Hazard ratio	95% CI of ratio	*P* value
Macrophages M1	0.0015	[0.000; 1.201]	0.0487
T cells CD4 naive	903.3076*E*+030	[0.000; 1.6002*E*+072]	0.099
Dendritic cells resting	0.0409	[0.000; 71.715]	0.4017
T cells CD4 memory activated	0.0002	[2.395*E*-009; 10.202]	0.1213
T cells follicular helper	0.0088	[0.000; 746.477]	0.4139
Eosinophils	871744005.3988	[92.062; 8.255*E*+015]	0.0120
Mast cells activated	3240.9197	[14.439; 727455.403]	0.0034
Mast cells resting	0.0013	[0.000; 37.612]	0.2044
Dendritic cells activated	3301.9673	[0.208; 52456610.539]	0.1007
T cells CD8	0.0074	[0.000; 2.108]	0.0889
T cells CD4 memory resting	11.0261	[0.158; 770.711]	0.2680
Plasma cells	1.3321	[0.025; 72.337]	0.8881
B cells naive	0.0013	[0.000; 138.9808]	0.1960
Macrophages M0	6.4783	[0.719; 58.367]	0.0957
Monocytes	0.3181	[3.12*E*-018; 32.34*E*+015]	0.9543
Neutrophils	624.5481	[0.0003; 1.17*E*+009]	0.3824
NK cells resting	147.3317	[0.0013; 16784367.328]	0.4007
Macrophages M2	0.0779	[0.0002; 35.724]	0.4144
B cells memory	6.2027	[2.83*E*-13; 135.8827*E*+012]	0.9099
T cells gamma delta	0.0000	[5.415*E*-021; 89.2*E*+009]	0.5586
NK cells activated	0.0748	[5.725*E*-009; 97716.806]	0.7539
T cells regulatory (Tregs)	0.0000	[5.8221*E*-011; 16.447]	0.1087

## Data Availability

Data supporting the results of the study can be available by emailing the first author or corresponding author.
